# Artificial Intelligence-based MRI Images for Brain in Prediction of Alzheimer's Disease

**DOI:** 10.1155/2021/8198552

**Published:** 2021-10-19

**Authors:** Xiaowang Bi, Wei Liu, Huaiqin Liu, Qun Shang

**Affiliations:** ^1^Department of Radiology, Zibo Central Hospital, Zibo 255000, Shandong, China; ^2^China-Israel fMRI Precision Neuroimaging Joint Laboratory, Zibo 255000, Shandong, China

## Abstract

The study aimed to explore the accuracy and stability of Deep metric learning (DML) algorithm in Magnetic Resonance Imaging (MRI) examination of Alzheimer's Disease (AD) patients. In this study, MRI data of patients obtained were from Alzheimer's Disease Neuroimaging Initiative (ADNI) database (A total of 180 AD cases, 88 women, 92 men; 188 samples in healthy conditions (HC), including 90 females and 98 males. 210 samples of mild cognitive impairment (MCI), 104 females and 106 males). On the basis of deep learning, an early AD diagnosis system was constructed using CNN (Convolutional Neural Network) and DML algorithms. Then, the system was used to classify AD, HC, and MCI, and the two algorithms were compared for the accuracy and stability of in classification of MRI images. It was found that in the classification of AD and HC, the classification accuracy and sensitivity of the deep measurement learning model are both 0.83, superior to the CNN model; in terms of specificity, the classification specificity of the DML model was 0.82, slightly lower than that of the CNN model; and that in the classification of MCI and HC, the classification accuracy and sensitivity of the DML model was 0.65, superior to the CNN model; and in terms of specificity, the classification specificity of the DML model was 0.66, slightly lower than that of the CNN model. It suggested that the DML model demonstrated better classification effects on early AD patients. The loss curve analysis results showed that, for classification of AD and HC or MCI and HC, the DML algorithm can improve the convergence speed of the AD early prediction model. Therefore, the DML algorithm can significantly improve the clarity and quality of MRI images, elevate the classification accuracy and stability of early AD patients, and accelerate the convergence of the model, providing a new way for early prediction of AD.

## 1. Introduction

Alzheimer's Disease (AD) is a chronic neurodegenerative cognitive disease. At the onset of the disease, patients will suffer from cognitive dysfunction such as memory loss and language function loss [1]. Nowadays, with the aging of the population, the AD population is increasing rapidly, and it has become a major disease threatening the health of the elderly, which seriously affects the quality of life of the elderly, and the need for nursing and care brings about heavy burdens to the patient's family and society [2]. Clinically, the cause of Alzheimer's disease is still unclear, and the condition is irreversible, and a thorough treatment of the disease has not yet been developed [3]. Only when AD is diagnosed in the early stage can it be possible to slow down or inhibit the progression. Thus, early prediction and diagnosis of AD is very important and meaningful in clinical treatment. Mild Cognitive Impairment (MCI) is a cognitive dysfunction between Alzheimer's disease (AD) and Healthy Controls (HC) [4]. Studies have found that, most patients with MCI have developed AD [5].

At present, Magnetic Resonance Imaging (MRI) technology is a main method to diagnose AD. Studies have discovered that, there are prominent biological signs in the brains of AD patients, which is conducive to the early prediction and diagnosis of AD [6]. In-depth clinical research on AD has revealed that, family inheritance is an important cause of AD [7].

Artificial intelligence (AI) has developed rapidly in recent years, and AI technology has been widely used in the medical field [8]. Nowadays, machine learning (ML) or Deep Learning (DL) algorithms are always incorporated into MRI imaging [9], but the above methods all have limitations [10]. The machine learning algorithm analyzes the MRI image only after manually determining the area, but subjective factors will affect the subjectivity of the results [11]. Deep learning algorithms can automatically extract features of MRI images, but fails to interpret these features. As a result, it is difficult to identify biological features of AD [3]. Convolutional Neural Networks (CNN) is a kind of Feedforward Neural Networks with deep structure and convolution computation, which is one of the representative algorithms of deep learning and has the ability of representation learning. It can effectively reduce the dimension of a large amount of data into a small amount of data, while retaining image features, in line with the principle of image processing. Deep metric learning (DML) is a metric learning method. It is to learn a mapping from the original feature to the low-dimensional and dense vector space, so that the distance between objects of the same class is relatively close by using the commonly used distance function in the embedding space, while the distance between objects of different classes is relatively far.

In the study, the MRI data (There were 180 cases of AD, including 88 women and 92 men. There were 188 HC samples, including 90 females and 98 males. There were 210 samples of mild MCI, 104 females and 106 males) of patients were from the Alzheimer's Disease Neuroimaging Initiative (ADNI) database. The traditional machine learning algorithms and Convolutional Neural Networks (CNNs) were optimized by deep learning to construct an early diagnosis system of AD based on Depth metric learning (DML) algorithm. The system was used to classify AD, MCI, and HC, and different algorithms were compared for the clarity and specificity of MRI images.

## 2. Materials and methods

### 2.1. Experimental data

The experimental data of this study were from the ADNI database [12]. The MRI image data used in this article were divided into 3 categories, namely: 180 cases of AD, including 88 cases of females, and 92 cases of males; 188 samples of HC, including 90 cases of females and 98 cases of males; and 210 samples of MCI, including 104 females and 106 males. There was no significant difference in age and gender of the three types of subjects, and the average age was approximately 74 years old.

### 2.2. Pre-processing of MRI images

Figure 1 showed the preprocessing of the MRI image, including correction, segmentation, template formation, and skull removal. The MRI images were obtained at various angles due to the head movement during MRI scan. Generally, the brain MRI image includes the skull and neck bones, and the skulls and neck bones are different in size, thickness, and length between individuals. The classification of AD is mainly to analyze the internal tissue structure of the brain, and thus the skull and neck bones in the MRI image are all noise signals.

### 2.3. CNN model and parameters

CNN is extensively used in the field of image recognition for its unique structure [13]. To use deep learning technology to automatically segment MRI images can greatly reduce the dependence on the subjective judgment of doctors. The traditional CNN structure mainly includes the convolutional layer, the pooling layer, and the fully connected layer. The neural unit layers of various functions are stacked to form a deep CNN, as shown in Figure 2. There are a total of 8 convolutional layers, and the size of the convolution kernel used by each convolutional layer is 3×3×3, and the step size is 1×1×1. There are 5 pooling layers, all pooling layers use Maximum pooling, and the core size and step size of the first pooling layer are 1×2×2, that is, the time dimension is not pooled, and the core size and step size of the remaining pooling layers are 2×2×2. There are two fully connected layers, and the length of the output column vector is 4096. There is a softmax layer. The convolutional pooling layer aims to reduce the size of the feature map by half and double the number of channels.

### 2.4. DML loss function

The classification data used in this study contained data of AD, HC, and MCI. They were classified into two categories, namely AD and HC, MCI and HC. In the classification of AD and HC, the category label of AD is 0 and the category label of HC is 1. In MCI and HC, the category label of MCI is 0 and the category label of HC is 1.

#### 2.4.1. Cross entropy loss function

This study uses the cross-entropy loss function, and the two-category cross-entropy loss function is adjusted to the following equation (1).

(1) $$\begin{array}{c} \text{cross}\_\text{entropy}=\frac{1}{N}\sum_{k=1}^{N}-\left[w_{k}\text{ln}x_{k}+\left(1-w_{k}\right)\text{ln}\left(1-x_{k}\right)\right], \end{array}$$

Where *N* refers to the batch size, *w*_*k*_ represents the category of the Kth subject, and *x*_*k*_ refers to the probability that the Kth category label predicted by the detection system is 1, calculated as follows.

(2) $$\begin{array}{c} x_{k}=\text{Softmax}\left(w_{k}\right)=\frac{\text{exp}\left(w_{k}^{1}\right)}{\exp\left(w_{k}^{0}\right)+\text{exp}\left(w_{k}^{1}\right)}, \end{array}$$

Where *w*_*k*_ refers to Kth classification vector, *w*_*k*_^0^ represents the first *w*_*k*_ value, and *w*_*k*_^1^ refers to the second *w*_*k*_ value.

#### 2.4.2. Loss function based on metric learning

The loss function of metric learning is expressed as equation (3).

(3) $$\begin{array}{c} {\text{loss}}_{\text{contrastive}}=\frac{2}{N\left(N+1\right)}\sum_{h=1}\sum_{g=h}\left[w_{hg}m\left(x_{h},x_{g}\right)+\left(1-w_{hg}\text{max}\left(a-D\left(x_{h},x_{g}\right)\right.,\;0\right)\right], \end{array}$$

Where *N* refers to the batch size, *a* refers to the interval, *x*_*h*_ is the *h*th sample and  *x*_*g*_ is the *g* th sample. When *x*_*h*_ and *x*_*g*_ belong to different categories, *w*_*hg*_ is 0; and when *x*_*h*_ and *x*_*g*_ belong to the same category, *w*_*hg*_ is 1. *D*(*x*_*h*_, *x*_*g*_) is calculated as equation (4), and *f*(*x*) represents the output vector.

(4) $$\begin{array}{c} D\left(x,y\right)=f\left(x\right)-f{\left(y\right)}_{2}. \end{array}$$

#### 2.4.3. Overall loss function

This research combines AD classification and DML to construct a DML loss function, expressed as follows.

(5) $$\begin{array}{c} \text{loss}={\text{cross}}_{\text{entropy}}+q\;{\text{loss}}_{\text{conrastive}}, \end{array}$$

Where cross_entropy_ is calculated by equation (1); and loss_conrastive_ is calculated by equation (3). The value of *q* is greater than 0, and it refers to the adjustment coefficient of classification and measurement loss.

### 2.5. Evaluation Index

The performance of predictive classification algorithms of early AD was evaluated factoring into Accuracy (Acc), Sensitivity (Sens), and Specificity (Spec). The number of patients accurately diagnosed is represented by the letter A, the number of normal subjects diagnosed as normal is represented by the letter B, the number of normal subjects who are incorrectly diagnosed as patients is represented by the letter C, and the number of patients who are mistakenly diagnosed as normal people is represented by the letter D. The involved indexes are calculated as follows.

Acc refers to the proportion of the number of people who can be correctly predicted and classified, calculated as equation (6).

(6) $$\begin{array}{c} Acc=\frac{A+B}{A+B+C+D}. \end{array}$$

Sens refers to the ratio of the patients who are correctly detected to the total number of patients, calculated as equation (7).

(7) $$\begin{array}{c} \text{Sens}=\frac{A}{A+D}. \end{array}$$

Spec refers to the ratio of the correctly detected normal samples to the total number of normal people, calculated as equation (8).

(8) $$\begin{array}{c} \text{Spec}=\frac{B}{B+C}. \end{array}$$

### 2.6. Statistical analysis

Statistical analysis was performed using SPSS 24.0 software, expressed as mean ± standard deviation (‾x ± s). The count data were analyzed by *t* test, and *α*=0.05. *P*＜0.05 was the threshold for significance.

## 3. Results

### 3.1. Brain MRI features of AD patients

Figure 3 below showed MRI images of the brain of AD patients and normal people. In the MRI images of the brain of AD patients, brain atrophy was observed, which mainly occurred in the hippocampus, parahippocampal gyrus, and medial temporal lobes. At the same time, ventricles were dilated.

### 3.2. MRI images of AD patients based on CNN and DML algorithms

Figure 4 showed the MRI images of AD patients after processed by CNN and DML algorithms. Compared with MRI images processed by the CNN algorithm, MRI images processed by DML algorithm had clearer texture and better imaging effects on cerebral blood vessels. Further, the sharpness was higher, so DML can greatly improve the visual sharpness of MRI images.

### 3.3. Comparison of classification results

CNN and DML models classified the patients separately, and they were compared for the classification accuracy, sensitivity, and specificity. The specific classification effects of AD and HC, MCI and HC were shown as below.

#### 3.3.1. Classification of AD and HC

Figure 5 below showed the classification results of AD and HC. It was noted that the classification accuracy and sensitivity of the deep measurement learning model are both 0.83, superior to the CNN model. In terms of specificity, the classification specificity of the DML model was 0.82, slightly lower than that of the CNN model.

#### 3.3.2. Classification results of MCI and HC

Figure 6 showed the classification effects of MCI and HC. It was noted that in terms of accuracy and sensitivity, the classification accuracy and sensitivity of the DML model was 0.65, superior to the CNN model; and in terms of specificity, the classification specificity of the DML model was 0.66, slightly lower than that of the CNN model.

### 3.4. Loss curve analysis

The convergence curves of the CNN model and the MDL model were analyzed, and the loss curves of AD and HC, MCI and HC were shown below.

#### 3.4.1. Classification of AD and HC

Figure 7 showed the loss curves of the classification of AD and HC when the CNN model and the DML model were used for training. It was noted that when the CNN model was used for training, as the number of iterations increased, the training loss decreased. At the beginning, the training loss decreased rapidly, but after 3000 iterations, the training loss decreased slowly, and the training loss tended to be stable and the model fully converged after 6000 iterations. When the DML model was used for training, the training loss decreased as the number of iterations increased. At the beginning, the training loss dropped quickly. After 2000 iterations, the training loss decreased slowly. The training loss tended to be stable and the model fully converged after 4500 iterations. Taken together, the DML model can improve the convergence speed of the model.

#### 3.4.2. Classification results of MCI and HC

Figure 8 showed the loss curves of the classification of MCI and HC when the CNN model and the DML model were used for training. It was noted that when the CNN model was used for training, as the number of iterations increased, the training loss decreased. At the beginning, the training loss decreased rapidly, but after 4000 iterations, the training loss decreased slowly, and the training loss tended to be stable and the model fully converged after 7000 iterations. When the DML model was used for training, the training loss decreased as the number of iterations increased. At the beginning, the training loss dropped quickly. After 3000 iterations, the training loss decreased slowly. The training loss tended to be stable and the model fully converged after 4500 iterations. Taken together, the DML model can improve the convergence speed of the model.

## 4. Discussion

AD is a chronic degenerative cognitive disease of the nervous system. At the onset of the disease, patients will suffer from cognitive dysfunction such as memory loss and language function loss. The disease has a long incubation period and will worsen with time [14]. The pathogenesis of AD still remains unclear, and it cannot be cured once diagnosed. Therefore, early diagnosis and prediction become particularly important. Only when AD is diagnosed in the early stage can it be possible to slow down or inhibit the progression [15]. In recent years, there is a large amount of research on the classification and prediction of early AD using traditional machine learning methods [16], and the classification and prediction of early AD using deep learning technology is a common occurrence [17]. For example, Folego et al. (2020) [18] used CNNs to process MRI images, and the classification accuracy of AD and HC reached 0.97. Perezn et al. (2019) [19] connected multiple image blocks to classify the MRI samples in the ADNI database, and the accuracy rate can reach 0.95. Therefore, to construct a simple, stable, and accurate early diagnosis system for AD is important for early intervention and treatment of AD. In order to explore the role of artificial intelligence in the prediction of early AD from MRI images, the CNN model and the DML model were used to classify AD, HC, and MCI.

Takenoshita et al. (2019) [20] extracted features of MRI samples in the ADNI database to classify AD, MCI, and HC, and the effect was very good. MRI of healthy persons and AD patients were compared, and it was found that brain atrophy occurred in AD patients, mainly in the hippocampus, parahippocampal gyrus, medial temporal lobe, and other brain regions, and ventricular dilation was also observed, which indicated that MRI images could clearly show the lesions in the brain domain of patients, and had diagnostic value. The classification accuracy and sensitivity of DML model were both 0.83, higher than those of CNN model. The classification specificity of DML model was 0.82, slightly lower than that of CNN model. Usually, sensitivity refers to the proportion of patients who are correctly diagnosed. If an AD patient is mistakenly diagnosed as a normal person, the opportunity for treatment will be missed and it will lead to serious consequences; if a normal person is mistakenly diagnosed as an AD patient, usually, he will be diagnosed again. Therefore, in clinical practice, specificity can be appropriately reduced to improve the sensitivity of prediction. Above, the DML model demonstrated better classification effects on early AD patients.

The training loss of CNN model decreased with the increase of iterations. After 3000 iterations, the decline rate of training loss tended to be gentle, and converged completely after 6000 iterations. The DML model also saw a decline in training loss with the increase of iterations. After 2000 iterations, the decline rate of training loss tended to be stable, and it completely converged after 4500 iterations. This showed that compared with the CNN model, the DML model in this study had a faster convergence speed and better computing performance. Figure 8 showed the loss curves of the classification of MCI and HC when the CNN model and the DML model were used for training. It was noted that when the CNN model was used for training, as the number of iterations increased, the training loss decreased. At the beginning, the training loss decreased rapidly, but after 4000 iterations, the training loss decreased slowly, and the training loss tended to be stable and the model fully converged after 7000 iterations. When the DML model was used for training, the training loss decreased as the number of iterations increased. At the beginning, the training loss dropped quickly. After 3000 iterations Whitwell, the training loss decreased slowly. The training loss tended to be stable and the model fully converged after 4500 iterations. Taken together, the DML model can improve the convergence speed of the model. Hence, the DML model can speed up the convergence for the classification of the both categories, which was in line with the research results of Vaithinathan et al. (2019) [21].

## 5. Conclusion

In the study, the MRI data used were from the ADNI database. On the basis of deep learning, an early diagnosis system for AD was constructed using CNN and DML algorithms. Then, the system was used to classify AD, HC, and MCI, and the two algorithms were compared for the accuracy and stability of in classification of MRI images. It was found that the DML algorithm can significantly improve the clarity and quality of MRI images, elevate the classification accuracy and stability of early AD patients, and accelerate the convergence of the model, providing a new way for early prediction of AD. However, some limitations in the study should be noted. The sample size is small, which will reduce the power of the study. In the follow-up, an expanded sample size is necessary to strengthen the findings of the study.

## Figures and Tables

**Figure 1:** Preprocessing of MRI images.

**Figure 2:** CNN structure.

**Figure 3:** MRI images of normal people and AD patients.

**Figure 4:** MRI images of AD patients processed by CNN and DML algorithms. *Note.* Figure 4A was an MRI image of AD patients based on CNN algorithm; and Figure 4B was an MRI image of AD patients based on DML algorithm.

**Figure 5:** Classification effects of AD and HC.

**Figure 6:** Comparison of classification effects between MCI and HC.

**Figure 7:** Loss curves of classification of AD and HC.

**Figure 8:** Loss curves of classification of MCI and HC.

## Data Availability

The data used to support the findings of this study are available from the corresponding author upon request.
